This article has been retracted.

# Regulatory Role of Zinc in Allergic Rhinitis through the IL-33/ST2 Pathway

**DOI:** 10.1155/2022/3718317

**Published:** 2022-01-07

**Authors:** Wulin Wen, Fengxia Yang, Xueliang Shen, Ningyu Feng, Huiyu Ha, Ruixia Ma

**Affiliations:** ^1^Department of Otolaryngology Head and Neck Surgery, Second Affiliated Hospital of Ningxia Medical University, The First People's Hospital of Yinchuan, Ningxia 753000, China; ^2^Department of Otolaryngology Head and Neck Surgery, The Third People's Hospital of Yinchuan, Ningxia 753000, China; ^3^Department of Otolaryngology Head and Neck Surgery, General Hospital of Ningxia Medical University, Ningxia 753000, China

## Abstract

**Objective:**

We aimed to investigate the expression of serum zinc and cytokines interleukin- (IL-) 13 and IL-33 in patients with allergic rhinitis (AR) and observe the effects of zinc on cytokines and pathway proteins in P815 mast cells stimulated by Artemisia annua allergen (Art.) in the IL-33/suppression of the tumorigenicity 2 (ST2) pathway. We also aimed to explore the possible regulatory role of zinc in AR and provide new ideas to determine the etiology and treatment of AR.

**Methods:**

AR patients treated from March to September in 2018 were selected as the research participants, and 50 healthy people in the same period were selected as the control group. Serum samples of all patients were collected, and those of AR patients were tested for the presence of allergens. The expression of IL-13 and IL-33 was detected by performing an enzyme-linked immunosorbent assay, while the serum zinc level was detected by conducting an inductively coupled plasma mass spectrometry. The cell counting kit (CCK-8) was used to detect the proliferation of P815 mast cells, and western blot was used to detect the expression of ST2, p38, and p65 proteins.

**Results:**

A total of 92 AR patients were included in the study; of them, 52 had mild AR, while 40 had moderate AR. The primary allergen found in AR patients was Artemisia, and the positivity rate was 53.26%. The serum zinc ion level of AR patients decreased, and the expression of IL-13 and IL-33 increased. After Art. was used to treat P815 mast cells, the expression of IL-33 in the cell supernatant increased in a concentration-dependent manner, the expression of receptor ST2 increased, and the expression of downstream p38 and p65 proteins increased. However, after treatment with ZnSO_4_, the expression of IL-33 in the cell supernatant decreased, and the expression of ST2, p38, and p65 protein decreased.

**Conclusion:**

The serum zinc level of AR patients decreased. In the IL-33/ST2 pathway, ZnSO_4_ can reduce the hypersensitivity of mast cells induced by Art.

## 1. Introduction

Allergic rhinitis (AR) is a group of allergic diseases with nasal symptoms as the primary symptoms, which can have several complications and has a complex pathogenesis. In recent years, the global AR incidence rate is increasing, affecting 40% of the population [1–4]. Therefore, a safe and effective treatment must be developed for an in-depth study of AR pathogenesis.

As a necessary type of mineral, zinc is widely involved in various functions of the human body [5]. Zinc deficiency is a risk factor for asthma [6, 7], with high risk, particularly in children with allergic diseases [8]. The high expression of interleukin (IL-4) in AR patients is related to low serum zinc levels [9]. In recent years, studies have shown that the IL-33/suppression of the tumorigenicity 2 (ST2) signaling pathway plays an important role in mast cell-mediated allergic diseases [10, 11]. As an endogenous “alarm hormone,” IL-33 plays a dual role (a cytokine and a nuclear factor) [12]. Although IL-33 participates in the growth and development of AR [13, 14], studies examining the role of IL-33 and zinc in the pathogenesis of AR are limited. Hence, this study aimed to investigate the possible regulatory effect of zinc on AR in the IL-33/ST2 pathway.

## 2. Materials and Methods

From March to September 2018, 92 AR patients [15] were selected as the research participants. According to the criteria proposed by Vanhoecke et al. [16], AR patients were divided into a mild group and moderate and severe group. At the same time, 50 healthy people (25 men and 25 women) were selected as the control group, and their age ranged from 4 to 60 years.

Approximately 5 ml of peripheral venous blood was obtained from all research participants, which was allowed to stand at room temperature for 1 hour; the serum was separated and aliquoted and stored at −80°C for later use. The administration of antihistamines, corticosteroids, and immunosuppressants was discontinued one week prior to blood collection.

### 2.1. Allergen Testing

AR patients were tested for serum allergens. There were 18 kinds of allergens; inhalant allergens include Artemisia, tree pollen (cypress, elm, willow, oak, birch, maple, walnut, Chinese parasol, and poplar), household dust mites, dog hair, cat hair, amaranth, mulberry, mold (*Penicillium punctatum*/*Mycoderma*/*Aspergillus fumigatus*/*Aspergillus niger*), and cockroaches; food allergens include chicken egg white, milk, shrimp, shellfish, crab, beef, cashew, mango, and pineapple. The results were divided into 7 grades: 0, none (0.00–0.34 IU/ml); 1, low (0.35–0.69 IU/ml); 2, increase (0.70–3.49 IU/ml); 3, significant increase (3.50–17.49 IU/ml); 4, high (17.50–49.9 IU/ml); 5, high (50.0–100.0 IU/ml); and 6, extremely high (>100 IU/ml).

### 2.2. Determination of Serum Zinc Levels by Inductively-Coupled Plasma Mass Spectrometry

The laboratory supplies used were stored in strong acid overnight to eliminate the residual trace elements and then cleaned with deionized water for standby. Four blank control groups with only mixed acid were set up, and the experiment was completed in the following order: sample addition, acid driving, constant volume, standard matching, and detection.

### 2.3. Statistical Analysis

All data were given in the form of means and standard deviations. Student's *t*-test was used to make comparisons. SPSS 20.0 software was used for all statistical analyses (SPSS, Chicago, IL, USA). *P* < 0.05 was statistically significant.

## 3. Experimental Results

A total of 92 AR patients were included in this study, of whom 43 were men and 49 were women. Over 52 patients had mild cases, while 40 had moderate and severe cases. No significant difference was observed in disease condition between patients with different genders or age ranges (Table 1).

Table 2 shows that the main allergen of AR is Artemisia, and the positivity rate is 53.26%. Among the study participants, 50 (54.35%) were allergic to more than three kinds of allergens.

The serum levels of IL-13 and IL-33 were 6.90 ± 5.34 and 15.64 ± 6.78 pg/ml in mild AR patients and 13.07 ± 2.89 and 23.62 ± 7.49 pg/ml in moderate to severe AR patients, respectively. Compared with the control group (3.43 ± 2.94 and 6.91 ± 4.87, respectively), the difference was significant (*P* < 0.05) (Figure 1).

The serum zinc levels in the mild and moderate-to-severe AR patients were 830 and 850 *μ*g/L, respectively. No significant difference was observed between the two groups. However, the difference was significant compared with the serum zinc level of 960 *μ*g/L in the control group (*P* < 0.05) (Figure 2).

With the increase of ZnSO_4_ concentration (50–300 *μ*mol/L), the proliferation of P815 mast cells increased significantly. At 12 h, when the concentration of ZnSO_4_ was 200 *μ*mol/L, cell proliferation was most noticeable. Therefore, the ZnSO_4_ concentrations of 50, 100, and 200 *μ*mol/L were selected as the intervention concentrations for subsequent experiments (Figure 3).

After stimulating P815 mast cells with Art. at concentrations of 0.01 and 0.1 µg/ml, the IL-33 expression increased (*P* < 0.05, *P* < 0.01). Subsequently, ZnSO_4_ treatment was initiated: (1) Compared with the blank control group A, the expression of IL-33 in group B, group C, group D, and group F decreased, which was significant (*P* < 0.05); the expression of IL-33 in group E increased, which was also significant (*P* < 0.05). (2) When the Art. concentration was fixed at 0.01 *μ*g/ml, compared with group B, the expression of IL-33 in group C and group D showed a downward trend, with no statistical significance; when the ZnSO_4_ concentration was fixed at 100 µmol/L, compared with group C, the expression of IL-33 in group E increased, with statistical significance (*P* < 0.05) (Figure 4).

When Art. stimulated the P815 mast cells, compared with the blank control group, the expressions of ST2, p38, and p65 increased in each group, and the difference in ST2 was not significant. Subsequently, ZnSO_4_ treatment was initiated: (1) Compared with the blank control group A, the expression of ST2 and p38 protein in each group decreased, while the expression of p65 decreased in groups C and F and increased in groups B, D, and E, but no significant difference was observed. (2) When the concentration of Art. was fixed at 0.01 *μ*g/ml, compared with group B, the expression of ST2, p38, and p65 in groups C and D decreased; when the concentration of ZnSO_4_ was fixed at 100 *μ*mol/L, compared with group C, the expression of ST2 and p65 increased, while the expression of p38 decreased in groups E and F, the difference in all of which was not significant (Figure 5).

## 4. Discussion

Pollen is the most common type of allergen that causes AR. This study found that the most common allergen is Art., which has no increasing trend compared with our research results 10 years ago [17]. In recent years, the allergy caused by Art. plants has attracted great public attention. We have actively taken a series of prevention and control measures, such as banning the planting of Art. green belt in this area and actively promoting the prevention before the allergy season.

We found that the expression of IL-33 in the serum of AR patients was increased, which was consistent with the results of other research [18–20]. There was a positive correlation between IL-33 in serum and the severity of AR in moderate-to-severe cases. As cytokines, IL-33 can induce the production of Th2 cytokines IL-4, IL-5, and IL-13 by binding with the ST2 receptor [21]. Moreover, the increased expression of IL-13 in the serum of AR patients may be related to the local inflammatory response of AR patients themselves and may be related to the production of Th2 cytokines promoted by IL-33.

Zinc deficiency is often associated with allergies [22], which plays an important role in stabilizing cell structure and maintaining cell function [4]. The level of trace element zinc in the serum of patients with AR decreased. ZnSO_4_ could promote the proliferation of mast cells at the condition of 50–200 *μ*mol/L, but it inhibited the proliferation when its concentration was higher than 300 *μ*mol/L. The high concentration of zinc may cause the imbalance of intracellular ions and lead to apoptosis. Previously, we found that the clinical symptoms of patients with zinc deficiency AR were significantly relieved by zinc supplementation [23]. Other studies have shown that higher zinc intake during pregnancy reduces the risk of postnatal asthma and eczema [24]. If there is excessive zinc in the tissue, the burden of liver and kidney function will increase, cell ultrastructure will be destroyed, and the immune function will be damaged [25, 26]. Therefore, zinc deficiency or excess can affect the proliferation, morphological changes, and immune function of cells. The effect of zinc on cell proliferation is related to its concentration and time. With the extension of experimental time and the increase of concentration, cell proliferation slows down and apoptosis occurs. Therefore, maintaining the dynamic balance of zinc plays an important role in preserving the immune function of cells. Thus, in clinical practice, patients with zinc deficiency are treated with zinc supplementation, and changes in the concentration of zinc ions must be monitored during the treatment to avoid excessive zinc.

In order to further understand the sensitization mechanism of Art. plants, after we used Art. to treat mast cells, the expression of IL-33 in the cell supernatant increased in a concentration-dependent manner, the expression of its receptor ST2 increased, and the expression of downstream p38 and p65 proteins increased. Therefore, Art. can sensitize P815 mast cells. When ZnSO_4_ and Art. were combined to intervene the mast cells, the expression of IL-33 decreased, and the expression of its ST2 protein and downstream p38 and p65 proteins decreased; when the concentration of Art. was fixed at 0.01 *μ*g/ml, the higher the concentration of ZnSO_4_, the more obvious the inhibition of this reaction; and when the concentration of ZnSO_4_ was fixed at 100 *μ*mol/L, with the increase of the concentration of Art., its inhibitory effect on allergic reaction also weakened. Therefore, the administration of ZnSO_4_ inhibited the allergic reaction to a certain extent, which was closely related to the expression of allergens and the intervention concentration of zinc. Hence, the key to AR intervention is to reduce the exposure to allergens and their accumulative actions to the greatest extent and to administer zinc reasonably and timely.

## 5. Conclusions

In conclusion, the serum zinc level of patients with AR decreased, and the expression of inflammatory cytokines increased. Zinc supplementation can relieve the allergic state. The clinical contributions of our study are as follows: (1) dynamic equilibrium of zinc is critical for maintaining cell immunological function. (2) In clinical practice, individuals with zinc insufficiency should be administered with zinc supplementation, and variations in zinc concentration are routinely monitored during therapy to avoid excessive zinc.

## Figures and Tables

**Figure 1:** Expression of IL-13 and IL-33 in the serum of AR patients and the control group. Compared with the control group, ^∗∗^*P* < 0.01.

**Figure 2:** Serum zinc levels of patients in the AR group and control group. Compared with the control group, ^∗∗^*P* < 0.01.

**Figure 3:** CCK-8 experiment detecting the proliferation of P815 mast cells 12 h after stimulation with different concentrations of ZnSO_4_ (*n* = 5).

**Figure 4:** (a) The expression of IL-33 in the supernatant of mast cells stimulated by Art. for 12 h; (b) the expression of IL-33 in the supernatant of mast cells treated by ZnSO_4_ combined with Art. for 12 h. ^∗^*P* < 0.05 and ^∗∗^*P* < 0.01. Group A: blank control group, group B: ZnSO_4_ 50 *μ*mol/L + Art. 0.01 *μ*g/ml, group C: ZnSO_4_ 100 *μ*mol/L + Art. 0.01 *μ*g/ml, group D: ZnSO_4_ 200 *μ*mol/L + Art. 0.01 *μ*g/ml, group E: ZnSO_4_ 100 *μ*mol/L + Art. 0.1 *μ*g/ml, and group F: ZnSO_4_ 100 *μ*mol/L + Art. 0.001 *μ*g/ml.

**Figure 5:** (a) The expression of ST2, p38, and p65 in mast cells stimulated by different concentrations of Art.; (b) the expression of ST2, p38, and p65 in mast cells treated by ZnSO_4_ combined with Art.; (c, d) the relative expression of ST2, p38, and p65 in groups A and B. ^∗^*P* < 0.05 and ^∗∗^*P* < 0.01. Group A: blank control group, group B: ZnSO_4_ 50 *μ*mol/L + Art. 0.01 *μ*g/ml, group C: ZnSO_4_ 100 *μ*mol/L + Art. 0.01 *μ*g/ml, group D: ZnSO_4_ 200 *μ*mol/L + Art. 0.01 *μ*g/ml, group E: ZnSO_4_ 100 *μ*mol/L + Art. 0.1 *μ*g/ml, and group F: ZnSO_4_ 100 *μ*mol/L + Art. 0.001 *μ*g/ml.

**Table 1:** Baseline data of AR patients.

	Mild	Moderate and severe	*χ* ^2^	*P*
Gender			0.016	0.898
Male	24	19		
Female	28	21		
Age			0.468	0.926
≤14 yrs	12	11		
15–29 yrs	13	11		
30–44 yrs	17	11		
45–59 yrs	10	7		

**Table 2:** Distribution of allergens in patients with AP.

Allergen	Grade							Positive number (*n*)	Positive rate (%)
	0	1	2	3	4	5	6		
Artemisia annua	0	0	20	19	6	3	1	49	53.26
Tree pollen	0	3	7	1	0	0	0	11	11.96
Mulberry	0	9	8	1	0	0	0	18	19.57
House dust mite	0	6	6	2	0	0	0	14	15.22
Amaranth	0	10	16	5	3	0	0	34	36.96
Cat dander	0	1	0	1	0	0	0	2	2.17
Dog dander	0	6	6	1	2	0	0	15	16.30
Mold	0	5	9	5	0	0	0	19	20.65
Cockroach	0	1	1	0	0	0	0	2	2.17
Egg white protein	0	6	4	0	0	0	0	10	10.87
Shellfish	0	7	1	0	0	0	0	8	8.70
Shrimp	0	3	2	0	0	0	0	5	5.43
Crab	0	5	2	1	0	0	0	8	8.70
Pineapple	0	7	1	0	0	0	0	8	8.70
Beef	0	3	1	0	0	0	0	4	4.35
Milk	0	3	1	0	0	0	0	4	4.35
Mango	0	5	6	2	0	0	0	13	14.13
Cashew nut	0	6	0	0	0	0	0	6	6.25
One allergen								25	27.17
Two allergens								17	18.48
≥3 allergens								50	54.35

## Data Availability

The datasets used and/or analyzed during the current study are available from the corresponding author on reasonable request.
